# Role of Folic Acid Drugs in the Treatment with Antithrombotic and Anticoagulant Drugs for Patients with Cardiovascular Diseases Based on the Analysis of Virtual Reality Medical Data

This article has been retracted.

**DOI:** 10.1155/2021/9914787

**Published:** 2021-08-04

**Authors:** Aiguo Zhang, Jing Wang, Qiang Jing

**Affiliations:** Pharmaceutical Department, The Fourth People's Hospital of Jinan, Jinan, Shandong 250031, China

## Abstract

In recent years, with the continuous progress and development of science and technology and the increasing maturity of medical technology, the incidence of cardiovascular diseases has gradually increased with the age of the population. In the case of cardiovascular disease, proper anticoagulant therapy can effectively prevent bleeding in the occurrence of events, so a more effective treatment of cardiovascular disease is considered a difficult problem to overcome. Therefore, this article proposes the role of folic acid drugs based on virtual reality medical data analysis in the treatment of cardiovascular disease patients with antithrombotic and anticoagulant drugs, in order to improve providing help for cardiovascular disease. This study selected patients with cardiovascular disease who were admitted to the hospital and extracted 100 patients with complete data and a one-year follow-up period, covering the overall status of the patients' cardiovascular risk factors, cardiovascular disease degree, and the occurrence of major cardiovascular adverse events. During the follow-up period, we analyzed the specific status of major cardiovascular adverse events and the occurrence of bleeding events and compared and analyzed the effects of folic acid drugs on the treatment with antithrombotic and anticoagulant drugs in patients with cardiovascular disease. Experiments have proved that the differences in the degree of cardiovascular stenosis and the number of cardiovascular disease vessels in the four groups are statistically significant (*P* < 0.01). The degree of cardiovascular stenosis in group D was lighter than that in groups A, B, and C, and the number of cardiovascular lesions was also less than that in groups A, B, and C. The differences were statistically significant (*P* < 0.05). This indicates that folic acid can effectively treat cardiovascular stenosis, prevent cardiovascular disease, and then treat patients with cardiovascular disease with antithrombotic and anticoagulant drugs. It provides an important basis for accurate clinical diagnosis and treatment.

## 1. Introduction

With the development of urbanization and the improvement of people's living standards, the aging of the population has become more and more serious, which is also accompanied by a rapid increase in cardiovascular diseases. Relevant data show that the incidence of cardiovascular disease in China is as high as 40%. Among the cardiovascular drug treatments, antithrombotic and anticoagulant drug therapy occupies a high position, which can effectively prevent the occurrence of cardiovascular disease and improve cardiovascular disease. The cure rate of the disease reduces the mortality rate of patients with cardiovascular diseases. In most cases, data centers in traditional hospitals are operated independently using multiple application systems. As system usage and scale grows, over time, equipment, operation, and maintenance costs increase, making it impossible to meet the high performance, high availability, and security requirements of information system data. However, virtual reality and cloud computing technologies can effectively solve these problems and provide powerful and important support for the analysis of medical data.

Antithrombotic/anticoagulant treatment for cardiovascular disease overseas is much faster than in China, and the development and renewal of antithrombotic/anticoagulant treatment technology for cardiovascular disease is progressing rapidly. Antithrombotic and anticoagulant treatments and treatments for cardiovascular disease have been significantly improved and developed. It is believed that the use of folic acid drugs to treat cardiovascular diseases will become an important breakthrough in the near future. Fernández-Montero et al. concluded that new oral anticoagulants have a relatively lower important bleeding risk. In terms of effectiveness, the recurrence rate of thrombosis after treatment with new anticoagulants is undoubtedly not inferior to warfarin, and it has not been seen to significantly increase the risk of bleeding, except for gastrointestinal bleeding [1]. Leone et al. used a heparin coating method based on hyaluronic acid. Clinical studies have shown that the coating method has better effects and less inflammatory response and can safely reduce the amount of heparinized heparin throughout the body during cardiopulmonary bypass [2]. Klingel et al. proposed to extend the anticoagulation time while reducing the recurrence of the disease, while the incidence of major bleeding increased by more than 3 times, of which the gastrointestinal tract is the most common bleeding site [3].

The use of folic acid drugs for the treatment with antithrombotic and anticoagulant drugs for cardiovascular disease began in Western countries. Compared to Western countries, my country's antithrombotic and anticoagulant treatment technologies for cardiovascular disease begin in the second half of clinical practice and their development is relatively slow. With the continuous progress and development of modern science and technology and the increasing maturity of medical technology, the use of folic acid drugs to treat cardiovascular diseases will be an important research work. Joo et al. studied the morphology, adhesion, and proliferation of cells on PVC pipes with different coatings. For the coating of cell adhesion, it is mainly determined by the uniformity of the coating rather than the coating material [4]. Leiter et al. used a photochemical fixation method to covalently bond dipyridamole to the polyurethane surface. It was found that dipyridamole significantly reduced the thrombus formation of the polyurethane surface and significantly reduced the adhesion of platelets, thereby improving the blood compatibility of the polyurethane [5]. Ozkan et al. pointed out that it is necessary to enhance the positive attitude of patients to treatment, reduce their anxiety, depression and other negative emotions, extend the survival period of cancer patients, improve their quality of life, and improve the recovery rate of patients; we believe that we will provide clinical standards for this illness [6–8].

This article mainly studies the role of folic acid drugs in the treatment with antithrombotic and anticoagulant drugs for patients with cardiovascular diseases based on virtual reality medical data analysis. Through the design of antithrombotic and anticoagulant drug treatment experiments for patients with cardiovascular diseases, the indicators of cardiovascular disease patients are analyzed at the same time, the logistic regression analysis method was used to correct various factors affecting recurring adverse cardiovascular events, and finally, the various test data of patients were analyzed [9, 10]. The innovations in this article not only pay attention to the role of folic acid in the treatment of patients with cardiovascular disease with antithrombotic and anticoagulant drugs, but also use virtual reality medical data analysis techniques to comprehensively and experimentally obtain experimental results. It is a systematic analysis that facilitates the treatment of cardiovascular disease processes and developmental research [11, 12].

## 2. Cardiovascular Disease and Antithrombotic and Anticoagulant Treatment

### 2.1. Image Processing

#### 2.1.1. Diffusion Tensor Imaging

Diffusion tensor imaging first assumes that the movement of molecules is a simple anisotropic diffusion process and calculates a representation of the diffusion tensor under the premise that the probability density function *p* satisfies a Gaussian distribution model with three variables of zero mean. The calculation method is shown in the following formula:

(1) $$\begin{array}{c} p\left(x\right)=G\left(x,Y,t\right). \end{array}$$

The Gaussian probability distribution function here is satisfied:

(2) $$\begin{array}{c} G\left(x,Y,t\right)={\left[{\left(4\pi t\right)}^{3}\det\left(Y\right)\right]}^{-\left(\frac{1}{2}\right)}\exp\left(-\frac{x^{T}Y^{-1}x}{4t}\right). \end{array}$$

Here, *Y* is the diffusion tensor and *t* is the diffusion time. If we transpose formula (1), we can get

(3) $$\begin{array}{c} A\left(q\right)=\exp\left(-tq^{T}Yq\right). \end{array}$$

If the logarithm of both sides of formula (3) is taken here at the same time, then a linear constraint on the unknown quantity *Y* expressed by *A*(*q*) can be obtained. Among them, the diffusion tensor *Y* can be written in the form of a matrix:

(4) $$\begin{array}{c} Y=\left[\begin{array}{ccc} Y_{xx} & Y_{xy} & Y_{xz}\\ Y_{yx} & Y_{yy} & Y_{yz}\\ Y_{zx} & Y_{zy} & Y_{zz} \end{array}\right], \end{array}$$

where *Y* is a symmetric positive semidefinite tensor; that is, there is always *Y*_*ij*_=*Y*_*ji*_ for all *i*, *j*=*z*, *y*, *z*. In order to obtain a complete evaluation value of the diffusion amount of a volume element, the average diffusion value is introduced as an invariant into the diffusion tensor imaging. It is an independent quantity that has nothing to do with the direction. It can measure the deviation of the uniform molecular motion on the surface of a body. Directly use the trace of the diffusion tensor *Y* to directly represent the diffusion mean *M*_*Y*_, and the calculation method is as follows:

(5) $$\begin{array}{c} M_{Y}=\frac{tr\left(Y\right)}{3}.\\ =\frac{Y_{xx}+Y_{yy}+Y_{zz}}{3}. \end{array}$$

The average diffusion value will be lower in the ischemic area of the brain, which is of great significance to the clinical application of medicine. Calculating the diffusion mean requires a correct estimation of the diffusion tensor *Y*. Therefore, various sampling schemes and linear optimization methods are used to calculate the diffusion tensor *Y*. According to the diffusion tensor *Y*, *Y*_app_(*x*) can be used to represent the characteristic diffusion coefficient in the *x*(=[*x*_1_, *x*_2_, *x*_3_]) direction, and the calculation formula is as follows:

(6) $$\begin{array}{c} Y_{\text{app}}\left(x\right)=\sum_{i,j=1}^{3}Y_{ij}x_{i}x_{j}, \end{array}$$

where *x* is the unit vector, which satisfies the condition *xx*^*T*^=1.

The three most commonly used invariant indicators are relative anisotropy, anisotropy comparison value, and volume ratio. The definition of relative anisotropy is as follows:

(7) $$\begin{array}{c} RA=\sqrt{\frac{{\left(\lambda_{1}-\bar{\lambda }\right)}^{2}+{\left(\lambda_{2}-\bar{\lambda }\right)}^{2}+{\left(\lambda_{e}-\bar{\lambda }\right)}^{2}}{3\bar{\lambda }}}. \end{array}$$

Among them,

(8) $$\begin{array}{c} \bar{\lambda }=\frac{\left(\lambda_{1}+\lambda_{2}+\lambda_{3}\right)}{3}. \end{array}$$

The anisotropy comparison value is defined as follows:

(9) $$\begin{array}{c} FA=\sqrt{\frac{3}{2}}\sqrt{\frac{{\left(\lambda_{1}-\bar{\lambda }\right)}^{2}+{\left(\lambda_{2}-\bar{\lambda }\right)}^{2}+{\left(\lambda_{e}-\bar{\lambda }\right)}^{2}}{\left(\lambda_{1}^{2}+\lambda_{2}^{2}+\lambda_{3}^{2}\right)}.} \end{array}$$

Finally, the definition of body proportion is

(10) $$\begin{array}{c} VR=\frac{3\lambda_{1}}{{\bar{\lambda }}^{3}},\\ Y_{ij}\left(t\right)=\frac{1}{2t}\langle s_{i}s_{j}\rangle . \end{array}$$

Relative anisotropy is a unitized standard deviation, and it can also represent the ratio between the anisotropic part and the isotropic part of the diffusion tensor *Y*. The anisotropy comparison value measures the difference in the diffusion size of the diffusion tensor *Y* in different directions, and it can accurately summarize the degree of anisotropy diffusion [13, 14].

#### 2.1.2. Image Classification Based on Deep Convolutional Network

*(1) Relative Entropy.* Relative entropy is *KL* divergence, which is used to measure the difference between two probability distributions. It means that the distribution *q*(*x*) simulates the real distribution *p*(*x*) compared to the simulation *p*(*x*) with *p*(*x*), which requires additional information [15]. The calculation formula of the relative entropy is

(11) $$\begin{array}{c} KL\left(p\left\|q\right.\right)=-\int p\left(x\right)\ln\;q\left(x\right)\text{d}x-\left(-\int p\left(x\right)\ln\;p\left(x\right)\text{d}x\right). \end{array}$$

Because the status of *p*(*x*) and *q*(*x*) in the above formula is not equal

(12) $$\begin{array}{c} KL\left(p\left\|q\right.\right)\neq KL\left(q\left\|p\right.\right). \end{array}$$

If the values of *p*(*x*) and *q*(*x*) are slightly different, then *KL* is greater than zero. Only when *p*(*x*)=*q*(*x*), *KL* is equal to 0.

*(2)Cross-Entropy*. Assuming there are two distributions *p*(*x*) and *p*(*x*), their cross-entropy on a given sample set is defined as follows:

(13) $$\begin{array}{c} H\left(p,\;q\right)=-\int p\left(x\right)\ln\;q\left(x\right)\text{d}x. \end{array}$$

Cross-entropy is used to measure the similarity between two probability distributions. It represents the information needed to simulate the real distribution *p*(*x*) with distribution *q*(*x*).

*(3) Cross-Entropy Loss*. Definition of cross-entropy loss function is

(14) $$\begin{array}{c} CE\left(p,y\right)=\left\{\begin{array}{cc} -\log\left(p\right), & y=1,\\ -\log\left(1-q\right), & \text{others.} \end{array}\right. \end{array}$$

For convenience, use *p*_*t*_ instead of *p*; then,

(15) $$\begin{array}{c} p_{t}=\left\{\begin{array}{cc} p, & y=1,\\ 1-p, & \text{others.} \end{array}\right. \end{array}$$

Then, cross-entropy can be abbreviated as

(16) $$\begin{array}{c} CE\left(p,y\right)=CE\left(p_{t}\right),\\ =-\log\left(p_{t}\right) \end{array}$$

where *p* represents the probability, the value of *y* is 1 or −1, and the range of *p* is 0 to 1. In order to improve the problem of unbalanced class standard samples, some scholars have proposed weighted cross-entropy loss [16, 17]:

(17) $$\begin{array}{c} CE\left(p_{t}\right)=-a_{t}\log\left(p_{t}\right). \end{array}$$

*(4) Loss of Focus*. Although weighted cross-entropy can control the weight of positive and negative samples, it cannot control the weight of easy to classify and difficult to classify samples. So, there is the focus loss function:

(18) $$\begin{array}{c} FL\left(p_{t}\right)=-{\left(1-p_{t}\right)}^{\gamma }\log\left(p_{t}\right). \end{array}$$

Here, *γ* is called the focal length parameter, and *λ* ≥ 0 and (1 − *p*_*t*_)^*γ*^ are called the modulation coefficient.

### 2.2. Smart Medical

#### 2.2.1. Smart Medical Needs

The smart medical system uses a portable ubiquitous network, so that users no longer need to monitor physiological information at a designated location, which is of great significance to elderly patients who have difficulty moving. Moreover, some diseases require long-term monitoring to obtain their signs, such as sudden pauses in heartbeat. In these cases, long-term stable and uninterrupted monitoring is required. Long-term stable monitoring is also needed to prevent the irreversible trauma caused by sudden outbreaks to the human body [18, 19]. If long-term monitoring of the abovementioned patients can be achieved, it will not only dig out the deep-seated pathology of the patients to facilitate targeted treatment, but, at the same time, it is also very helpful for urgent treatment of diseases, because actually the best treatment period for these diseases is at the beginning of the outbreak. If the most beneficial treatment can be carried out on the patient at the first moment, the user's condition will be better. Realizing the monitoring of user's physiological information anytime and anywhere is an important part of modern medical treatment. Therefore, the proposal of smart medical treatment is also proposed by using the technological development of modern wireless communication and portable equipment [20, 21].

Respiration signals are also very beneficial to human health. This is because for a normal healthy subject, more than ten breathing processes are required under normal circumstances. In some tired and large exercise states, the human body's breathing will change. It is generally believed that the heart can complete four movements to complete a cycle of breathing, so the human body's breathing cannot be too fast or too slow. If the smart medical system considers that the user's video information needs to be transmitted to the smart medical diagnostic center under special circumstances, the portable terminal will start the video capture and transmission function [22, 23]. This function collects the user's video and audio signals through the camera and microphone system on the portable terminal. Then, the portable terminal transmits the collected audio and video signals to the smart medical storage and processing terminal for processing via the wireless network in a timely and fast manner [24].

#### 2.2.2. Smart Medical Construction Goals

The portable terminal is used to collect the physiological information of the human body, and the collected physiological information terminal system will be transmitted to the smart medical storage and processing terminal through the wireless network in the shortest time [25, 26]. The storage and processing system module will realize the real-time storage of the user's physiological information transmitted from each terminal, and the smart medical system will also display the physiological information of the human body in time, so that the doctor can view the physiological monitoring information of the user concerned in real time. The information transmission and data storage module mainly realizes the real-time transmission of the information collected by the portable terminal to the storage end of the intelligent medical system.

Considering that diseases such as heart disease are very sensitive to rescue time, the time delay between information collection, wireless transmission, and data storage must be taken into consideration when designing the information transmission and data storage function modules. At the same time, in order to facilitate the diagnostician to have a better grasp of the status of the patient, the main body visual video transmission function is turned on when necessary [27, 28]. The information collected by the mobile device is sent to the information storage, and the smart medical process is completed. This makes it possible to monitor the health of the human body. Smart medical processing enables real-time display of data collected on mobile devices and sends human physiological information to relevant diagnosticians via a smart medical system so that doctors can get real-time patient information as quickly as possible. You can quickly create diagnostic information. It helps to achieve timely rescue of the patient.

## 3. Experimental Design of Antithrombotic and Anticoagulant Drug Therapy for Patients with Cardiovascular Diseases

### 3.1. Test Subject

The trial selected 336 patients with cardiovascular disease admitted to a hospital from January to July 2019 and recorded the main adverse cardiovascular events and bleeding events of the patients in January, June, and one year after antiplatelet drug treatment. In this study, there were 107 patients with complete data and consistent follow-up time of 1 year. We selected 100 patients. The general information of these 100 patients is shown in Table 1. According to different antiplatelet treatments, it is divided into clopidogrel and aspirin dual-treatment group, clopidogrel group, aspirin group, and folic acid drug group. Analyze the overall situation of the patients' cardiovascular risk factors, the degree of cardiovascular disease, the occurrence of major adverse cardiovascular events, the specific situation of the major adverse cardiovascular events during the follow-up period, and the occurrence of bleeding events, and compare and analyze the antithrombotic effects of folic acid in patients with cardiovascular diseases and the role of anticoagulant therapy.

### 3.2. Test Method

All patients receive second-line preventive treatment for angiotensin-converting enzyme inhibitors, nitrates, statin lipid-lowering agents, *β*-receptor blockers, calcium channel blockers, and other standardized cardiovascular diseases, depending on their condition to select. Based on Group A, use aspirin 100 mg + clopidogrel 75 mg, given orally once daily; Group B, clopidogrel 75 mg orally once daily; Group C, aspirin 100 mg, orally administered once daily; and Group D, folic acid drug 100 mg, orally administered once daily. All patients were followed up for 1 year.

### 3.3. Observation Indicators

General clinical data and cardiovascular risk factors for patients with cardiovascular disease include age, smoking history, hypertension, diabetes, hyperlipidemia, length of disease, and degree of disease. Multivariate logistic regression analysis was used to adjust for various factors that influence the recurrence of major cardiovascular adverse events. Major cardiovascular adverse events during the 1-month, 6-month, and 1-year follow-up of antiplatelet drug treatment and bleeding complications after 1 year were recorded.

### 3.4. Statistical Processing

Statistical analysis was performed with SPSS 13.0 statistical software. The significance test of the difference was performed by one-way analysis of variance. The difference between the two groups was tested by LSD-*t*. The effect of folic acid on the treatment of cardiovascular disease patients with antithrombotic and anticoagulant drugs was performed by group *t*-test. *P* < 0.05 is considered to be statistically significant.

## 4. Antithrombotic and Anticoagulant Drug Therapy for Patients with Cardiovascular Diseases

### 4.1. Evaluation Index System Based on Index Reliability Testing

Here, we perform reliability analysis on all reliability indicators of each object, and the reliability indicators we choose for each object are slightly different. The results are shown in Table 2.

It can be seen from Figure 1 the overall situation of the patient's major adverse cardiovascular events, the specific situation of the major adverse cardiovascular events during the follow-up period, and the occurrence of bleeding events. The data obtained from various indicators have a very good effect on this experiment (*α* > 0.8); the data obtained from the patient's cardiovascular risk factors and the degree of cardiovascular disease have an acceptable impact on this experiment (*α* > 0.7), indicating that this article is studying the effects of folic acid in the cardiovascular system. The five indicators selected for the role of antithrombotic and anticoagulant drugs in the treatment of disease patients are reasonable, which provide a basis for subsequent continued experiments.

### 4.2. Evaluation Index System Based on Test Data

#### 4.2.1. Analysis Based on Cardiovascular Risk Factors

Here, we analyze the risk factors that cause cardiovascular disease and analyze the occurrence of different risk factors. The results are shown in Table 3.

As can be seen from Figure 2, Group A had 11 cases (44%) with a history of smoking, 17 cases (68%) with hypertension, 7 cases (28%) with diabetes, and 15 cases with high total cholesterol. 60% of patients had a low-density lipoprotein concentration of 4.14 mmol/L, while those with a low-density lipoprotein concentration higher than 1.8 mmol/L accounted for 80%. Group B had 9 patients (36%) with a history of smoking, 16 patients (67%) with hypertension, 7 patients (28%) with diabetes mellitus, 16 patients (60%) with total cholesterol exceeding 4.14 mmol/L, and 21 cases (84%) with low-density lipoprotein above 1.8 mmol/L. Group C had 10 patients (40%) with smoking history, 16 patients (64%) with hypertension, 9 patients (36%) with diabetes, 13 patients (52%) with total cholesterol above 4.14 mmol/L, 20 cases (80%) with low-density lipoprotein above 1.8 mmol/L, and 6 cases (24%) with a history of smoking. Group D had 10 cases (40%) with hypertension, 5 cases (20%) with diabetes, 9 cases (36%) with total cholesterol above 4.14 mmol/L, and 17 cases (68%) with low-density lipoprotein more than 1.8 mmol/L (68%). The four groups of patients had no difference in the statistical significance of smoking history, hypertension history, diabetes history, total cholesterol, and low-density lipoprotein (*P* > 0.05).

#### 4.2.2. Comparison of the Degree of Cardiovascular Disease

Here, we analyze the degree of cardiovascular disease and analyze the degree of cardiovascular disease in the patient according to the degree of cardiovascular stenosis and the number of diseased vessels. The results are shown in Tables 4 and 5.

As can be seen from Figure 3 and Table 4, the differences in the degree of cardiovascular stenosis and the number of cardiovascular disease vessels in the four groups were statistically significant (*P* < 0.01). The results of the pairwise comparison showed that the degree of cardiovascular stenosis in group D was lighter than that in groups A, B, and C, and the number of cardiovascular lesions was also lower than that in groups A, B, and C. The difference was statistically significant (*P* < 0.05). This shows that folic acid drugs are effective in treating cardiovascular stenosis and preventing cardiovascular disease.

#### 4.2.3. Multivariate Logistic Regression Analysis of Risk Factors for Major Adverse Cardiovascular Events

The risk factors of major adverse cardiovascular events in patients with cardiovascular diseases were analyzed. The results of the 1-year follow-up are shown in Table 6.

It can be seen from Figure 4 that smoking history, hypertension, and diabetes are risk factors for major adverse cardiovascular events in patients with cardiovascular disease. The OR values are 0.663, 0.546, and 0.179, respectively, which are all statistically significant (*P* < 0.05). High total cholesterol, high-low-density lipoprotein, number of diseased vessels, and degree of diseased vessel stenosis are not risk factors for recurring adverse cardiovascular events in patients with cardiovascular disease.

#### 4.2.4. Overall Situation of Major Adverse Cardiovascular Events

The overall situation of the major adverse cardiovascular events is analyzed here, and the results of the 1-year follow-up are shown in Table 7.

It can be seen from Figure 5 that the overall main adverse cardiovascular events of the four groups of patients were 28%, 40%, 36%, and 16%, and the differences were statistically significant (*P*=0.021 and *P* < 0.05). There was a statistically significant difference in the major adverse cardiovascular events between group D and groups A, B, and C (*P* < 0.05).

#### 4.2.5. Usage Rate of Proton Pump Inhibitors and Bleeding Events

Here, the use rate of proton pump inhibitors and the occurrence of bleeding events are analyzed, and the results are shown in Table 8.

It can be seen from Table 8 that the use rate of proton pump inhibitors in group A is 24%, that in group B is 8%, that in group C is 16%, and that in group D is 8%, and the difference is statistically significant (*P*=0.002, *P* < 0.01). After 1 year of follow-up, the incidence of bleeding events was 4% in group A, group B, and group C. There was no bleeding event in group D, and the difference was not statistically significant (*P*=0.433 and *P* > 0.05).

## 5. Conclusions

Currently, there is no standard monitoring method for assessing the anticoagulant effect of new anticoagulants. Even if they affect coagulation function, the relationship between these effects and bleeding and thrombosis has not been quantified. For drugs such as warfarin, which have a narrow therapeutic range, the anticoagulant effect should be monitored regularly for a long period of time in consideration of the safety of patient use. So far, there is no specific antagonist for complications such as bleeding caused by new oral anticoagulants. The degree of cardiovascular stenosis in group D was lighter than that in groups A, B, and C, and the number of cardiovascular lesions was also less than that in groups A, B, and C. The differences were statistically significant (*P* < 0.05). This shows that folic acid medicine has the effect of treating cardiovascular stenosis and preventing cardiovascular disease. The shortcoming of this study is that in the design stage of the study, it was not considered that different genders of patients may have different psychological endurance, which may have a certain impact on the results of psychological interventions and should be taken into consideration.

## Figures and Tables

**Figure 1:** Indicator reliability test analysis chart.

**Figure 2:** Cardiovascular disease risk factor analysis chart.

**Figure 3:** Analysis of the number of diseased vessels.

**Figure 4:** Multivariate logistic regression analysis chart of risk factors.

**Figure 5:** Analysis chart of the overall situation of major adverse cardiovascular events.

**Table 1:** General information of the two groups of patients.

Group	Number of cases		Years	Course of disease	Years of education
	Male	Female			
A	14	11	67.43 ± 6.42	127 ± 6.7	11 ± 3.12
B	17	8	68.62 ± 4.53	119 ± 9.4	11 ± 2.57
C	15	10	66.95 ± 8.16	130 ± 3.3	10 ± 4.38
D	17	11	67.84 ± 5.74	115 ± 11.2	11 ± 4.11

**Table 2:** Data sheet of evaluation index system for index reliability testing.

	Very clear	Clear	General	Not clear	Chaotic	Alpha
Cardiovascular risk factors	3.69	4.35	4.00	0.43	0.56	0.8662
Degree of cardiovascular disease	3.94	3.47	3.94	0.33	0.47	0.8754
Overall situation of adverse cardiovascular events	3.55	4.04	4.39	0.54	0.53	0.7831
Specific circumstances of adverse cardiovascular events during follow-up	3.53	3.47	4.50	0.75	0.34	0.7416
Occurrence of bleeding events	3.72	3.66	4.69	0.70	0.52	0.7364

**Table 3:** Cardiovascular disease risk factor data sheet.

Attributes	A (%)	B (%)	C (%)	D (%)	*T*	*P*
Smoking	11 (44)	9 (36)	10 (40)	6 (24)	2.453	0.280
High blood pressure	17 (68)	16 (64)	16 (64)	10 (40)	1.310	0.579
Diabetes	7 (28)	7 (28)	9 (36)	5 (20)	1.436	0.433
Total cholesterol	15 (60)	16 (64)	13 (52)	9 (36)	1.489	0.372
Low-density lipoprotein	20 (80)	21 (84)	20 (80)	17 (68)	0.479	0.751

**Table 4:** Cardiovascular stenosis data sheet.

Cardiovascular stenosis	A	B	C	D
Moderate	5	10	20	22
Severe	20	15	5	3

**Table 5:** Data sheet of diseased vessels.

Diseased vessels	A	B	C	D
1	12	15	19	21
2	6	5	5	4
3	7	5	1	0

**Table 6:** Multivariate logistic regression analysis of risk factors.

	SE	Wald	OR	*P*
Smoking	0.203	0.249	0.663	0.005
High blood pressure	0.194	0.823	0.546	0.001
Diabetes	0.175	0.191	0.179	0.001
Total cholesterol	0.196	0.070	0.831	0.089
Low-density lipoprotein	0.261	0.844	0.634	0.126
Diseased vessels	0.103	0.032	0.977	0.987
Cardiovascular stenosis	0.187	0.032	0.996	0.939

**Table 7:** Data sheet on the overall situation of major adverse cardiovascular events.

	A	B	C	D	*X* ^2^	*P*
Overall major adverse cardiovascular events	7	10	9	4	7.375	0.021
Death	0	1	1	0	5.406	0.061
Angina pectoris	6	7	7	2	3.543	0.076
Myocardial infarction	1	1	0	0	2.430	0.080
Stent stenosis	0	0	0	0	9.401	0.065

**Table 8:** Bleeding incident data sheet.

	A	B	C	D	*X* ^2^	*P*
Proton pump inhibitor	6	2	4	2	3.236	0.002
Bleeding event	1	1	1	0	1.610	0.433

## Data Availability

Data sharing is not applicable to this article as no datasets were generated or analyzed during the current study.
